# Biliary Drainage Reduces Intestinal Barrier Damage in Obstructive Jaundice by Regulating Autophagy

**DOI:** 10.1155/2022/3301330

**Published:** 2022-07-15

**Authors:** Xianfeng Zhang, Bojian Peng, Yuan Zhang, Yongjun Zhang, Xiushan Lu, Yanwen Cao

**Affiliations:** Department of Gastroenterology, Guangzhou Huadu District People's Hospital, Guangzhou, China

## Abstract

This study aims to investigate the mechanism by which biliary drainage reduces intestinal barrier damage in obstructive jaundice (OJ). A biliary drainage model was established in rats with OJ to detect changes in inflammatory factors and diamine oxidase (DAO), a marker of intestinal mucosal damage. The expression of autophagy-related genes in the intestinal mucosa after biliary drainage was detected using a reverse transcription-polymerase chain reaction. The rats were separated into two groups that received the autophagy activator rapamycin (RAPA) or the autophagy inhibitor 3-methyladenine (3-MA) to further investigate whether biliary drainage could alleviate the inflammatory response, oxidative stress, mitochondrial complex IV damage, and thus barrier damage in rats with OJ. The expression levels of inflammatory factors and the serum DAO content were increased in rats with OJ (*P* < 0.05). Biliary drainage further induced autophagy, reduced the expression levels of inflammatory factors, decreased the serum DAO content (*P* < 0.05), and improved intestinal mucosal damage. Administration of RAPA to OJ rats with biliary drainage increased autophagy (*P* < 0.05); decreased inflammatory factor secretion (*P* < 0.05), the serum DAO content (*P* < 0.05), oxidative stress (*P* < 0.05), and mitochondrial respiratory chain complex IV damage (*P* < 0.05); and ameliorated intestinal mucosal injury in OJ rats. When OJ rats were treated with 3-MA, intestinal mucosal injury, intestinal mitochondrial injury, and oxidative stress were all aggravated (*P* < 0.05). Biliary drainage can reduce the expression of inflammatory factors, oxidative stress, and mitochondrial injury by inducing intestinal mucosal autophagy in OJ rats, thus suggesting its role in the alleviation of intestinal mucosal injury.

## 1. Introduction

As a clinically common disease, obstructive jaundice (OJ) has a high probability of impairing the intestinal mucosal barrier and indirectly contributes to increased mortality [1]. The current recommended surgical approach to treat OJ is biliary obstruction relief [2], which mainly involves biliary intrahepatic and extrahepatic drainage. However, recent research has revealed that internal biliary drainage (BD) is superior to external BD [3], with some studies showing that internal BD is more effective in improving the intestinal barrier and reducing endotoxin absorption than external BD [4]. Intrahepatic BD was also shown to increase the number of cuprocytes, repair the mucosal layer, and restore the intestinal mucosal barrier [5]; however, the specific mechanism underlying these effects needs to be investigated further.

Intestinal epithelial cells are the most important component of the intestinal mucosal barrier [6]. Diamine oxidase (DAO) is widely expressed in the epithelial chromaffin cytoplasm of the intestinal mucosa. Chen et al. [7] revealed that intestinal mucosal cells release large amounts of DAO into the plasma in response to damage; therefore, an increase in the plasma DAO level can be used as a marker to confirm damage to the intestinal mucosa.

Autophagy is an intracellular degradation pathway that occurs under energy deficiency, hypoxia, pathogen infection, or stress in the body, which is crucial in maintaining cellular homeostasis [8]. Recent studies have shown a close relationship between the autophagy response in vivo with cardiovascular diseases, tumors, infections, and neurodegenerative diseases [9]. With a deepened understanding of autophagy, studies have also been conducted to determine the mechanism underlying its role in intestinal barrier dysfunction [10]. Autophagy has been shown to play a role in regulating the inflammatory response through a variety of mechanisms [11]. There is evidence that autophagy protects intestinal barrier function in patients with inflammatory bowel disease, primarily by modulating the tight junction proteins and inflammatory responses [12]. However, there are few studies on the role of autophagy in OJ, and it is unclear whether autophagy is involved in the pathology of OJ-induced intestinal barrier injury.

We hypothesized that autophagy is a crucial molecular biological mechanism involved in OJ-induced intestinal barrier injury, which can be mitigated by inhibiting autophagy through BD. To test this hypothesis, in this study, a rat model of OJ treated by BD was first constructed; rapamycin (RAPA) and 3-methyladenine (3-MA) were then administered to investigate whether BD could alleviate intestinal barrier injury by modulating autophagy.

## 2. Materials and Methods

### 2.1. Animals

Seventy male Sprague-Dawley rats (8–10 weeks of age, 250 g) were purchased from the Animal Experimental Center, and all rats were maintained at constant temperature and humidity with a 12-hour dark/light cycle. The rats had free access to adequate feed and water. This experiment was approved by the Animal Ethics Committee of our institute, and all animals were handled in strict accordance with the “Guidelines for the Protection and Application of Laboratory Animals” issued by the National Institute of Health.

### 2.2. Experimental Design

This experiment was divided into two parts. In Experiment 1, we explored whether autophagy occurs in the intestinal mucosa of OJ and whether it is promoted after BD treatment. The experimental animals were randomly divided into three groups by a random number table. All animals were numbered according to 1–30, then 30 numbers were transcribed from the random number table, each number was divided by 3, and 1, 2, and 3 represented the sham group, obstructive jaundice group (BDL group), and biliary drainage group (ID group). The results showed that 10 animals were classified into the sham group, 10 animals were classified into the BDL group, and 10 animals were classified into the ID group: the sham operation group (Sham group), where only an incision was made without common bile duct ligation; the obstructive jaundice group (BDL group), which involved common bile duct ligation; the internal bile drainage group (ID group), which involved both common bile duct ligation and internal BD surgery. In Experiment 2, we performed internal BD on the OJ rats, followed by treatment with an autophagy inhibitor or agonist, and observed the changes in autophagy in the intestinal mucosa of the OJ rats. Using a random number table, 40 experimental rats were divided into the OJ group that received common bile duct ligation (BDL group); the internal BD group (ID group) that received internal BD and common bile duct ligation; the autophagy agonist RAPA intervention group (IDR group) that involved common bile duct ligation and internal BD, followed by intragastric intervention with RAPA (2 mg/kg per day) 7 days after surgery; and the autophagy inhibitor 3-methyladenine intervention group (ID3-MA group) that involved common bile duct ligation and internal BD, followed by intragastric treatment with 3-methyladenine (24 mg/kg per day). A flowchart of the experimental design is shown in Figure 1.

### 2.3. Anesthesia

During the first operation, the rats were injected with 2% sodium pentobarbital intraperitoneally as anesthesia at 30 mg/kg.

During the second operation, different groups received a different anesthesia method. Experimental animals in the OJ and Sham groups were anesthetized by intraperitoneal injection of 2% pentobarbital (30 mg/kg body weight) to collect specimens. The experimental rats in the IDR and ID3-MA groups were given isoflurane inhalation as an anesthetic, and a mixture of 95% oxygen and 5% isoflurane was provided during the induction of anesthesia (gas flow rate of approximately 0.5 L/min) and during the operation to maintain anesthesia with 98% oxygen and 2% isoflurane mixed gas (flow rate of approximately 0.5 L/min).

During the third operation, the experimental rats in the ID, IDR, and ID 3-MA groups were anesthetized by intraperitoneal injection of 2% sodium pentobarbital (30 mg/kg) and specimens were collected.

### 2.4. Surgical Procedure

#### 2.4.1. OJ Model Establishment (BDL Group)

For the first operation, the rats were first weighed to determine the appropriate dose of anesthesia and 2% sodium pentobarbital was injected into the intraperitoneal cavity. Once anesthesia was successful, the skin was prepared following routine procedures, disinfected with iodophor, and bacteria plastic film and sterile gauze were spread over the surgical area. Starting from the xiphoid process, an incision was made layer by layer along the white line of the abdomen. The incision was approximately 1.2 cm long. After proper abdominal exposure, the duodenum was gently lifted from the pylorus with a hook to expose the bile ducts, and the exposed intestines were covered with wet gauze dipped in saline. The bile duct was carefully separated at the junction of the bile duct and the pancreas, and the bile duct was ligated twice. To prevent the bile duct from recanalizing, it was cut off by ophthalmic scissors between the two ligatures, and the duodenum was reset. The abdomen was closed layer by layer to create the OJ model. On the 8th day after the operation, the ileal tissue and blood samples were collected.

Morphine, paracetamol, and other analgesic drugs have a certain effect on autophagy, so we did not take related analgesic measures after surgery [13, 14]. All rats were killed by spinal cord dislocation, which met the requirements of animal ethics.

#### 2.4.2. Postoperative Monitoring

We monitored the wound healing of rats and observed whether there were signs of exudative infection every other day. It lasted until the rats completed the experiment and ended their lives.

#### 2.4.3. Sham Group

The rats were weighed before the first operation, and the appropriate dose of anesthesia was calculated. After a successful intraperitoneal injection of 2% pentobarbital sodium anesthesia, the operation area was routinely prepared, disinfected with iodophor, and spread with sterile plastic film and sterile gauze. The incision was made layer by layer along the white line of the abdomen, starting from under the xiphoid process. The incision was approximately 1.5 cm long. After proper abdominal exposure, the duodenum was gently lifted at the pylorus with a hook to expose the bile duct. The bile duct was carefully separated at the junction of the bile duct and the pancreas, the ligature was passed under the bile duct, and the knot was loosened but not closed; the bile duct was not cut off so that the bile remained unobstructed. The abdomen was closed layer by layer to make the sham model, and the ileal tissue and blood samples were collected on the 8th day after the operation.

#### 2.4.4. ID Group

The first operation was performed as described above for the OJ group, and the second operation was performed 7 days later. After successful gas inhalation anesthesia, routine skin preparation, and iodophor disinfection, aseptic plastic film and aseptic gauze were applied to the abdominal operation area. The last incision was made from the bottom of the xiphoid process. The incision was approximately 2.0 cm long. After proper abdominal exposure, the enlarged bile duct was exposed. A hook was used to carefully separate the bile duct and two 4–0 silk threads were passed under the bile duct. A 10 ml syringe was used to pierce the end of the bile duct to extract a small amount of bile. After removing the injection needle, one end of the drainage tube was quickly removed. The end of the enlarged bile duct was then inserted along with the needle port and fixed by double ligation to prevent the drainage tube from slipping off. The other end of the drainage tube was placed in the duodenum and embedded using a purse-string suture. The abdomen was closed to establish the ID model, and the ileal tissue and blood samples were collected on the 15th day after the operation.

#### 2.4.5. IDR Group

The first and second operations were the same as those described above for the establishment of the BDL model and ID group, and then the rats received rapamycin (2 mg/kg per day) administered in the stomach every other day from the 15th day after the operation until the 22nd day. The ileal tissue and blood samples were collected on the 22nd day.

#### 2.4.6. ID3-MA Group

The first and second operations were the same as those described above for the establishment of the BDL model and ID group. Starting from the 15th day after the second operation, the rats were administered 3-methyladenine every other day (24 mg/kg per day) via gavage, which continued until the 22nd day, and then the ileal tissue and blood samples were collected on the 22nd day.

### 2.5. Detection of Plasma Inflammatory Factors and DAO Using Enzyme-Linked Immunosorbent Assay (ELISA)

The levels of interleukin (IL) 6, IL-1*β*, DAO, and tumor necrosis factor (TNF)*α* in serum and ileum samples were determined using ELISA kits (Shanghai Enzymatic Biotechnology Co., Ltd., Shanghai, China).

### 2.6. Reverse Transcription-Polymerase Chain Reaction (RT-PCR)

TRIzol (Invitrogen, Grand Island, NY, USA) was used to homogenize the ileal mucosa (IM) tissues and extract RNA. cDNA was synthesized using a reverse transcription kit (MBI, USA). Multiple reactions were performed twice, and the intensity of the DNA bands was measured using Quantity One software (Bio-Rad, Hercules, CA, USA). The expression levels were standardized with reference to the internal control *β*-actin gene. Primers are shown in Table 1.

### 2.7. Measurement of Oxidative Stress Indicators

ELISA kits (Shanghai Beyotime Biotechnology Co., Ltd.) were used to determine the levels of glutathione (GSH), malondialdehyde (MDA), hydrogen peroxide (H_2_O_2_), and reactive oxygen species (ROS) in serum and ileum samples according to the manufacturer instructions.

### 2.8. Determination of Mitochondrial Respiratory Chain Complex Activity

The activity of mitochondrial respiratory chain complex IV in ileum samples was assessed using a complex kit (Shanghai Beyotime Biotechnology Co., Ltd.).

### 2.9. Statistical Analysis

Data are expressed as mean ± SEM. Statistical Product and Service Solutions (SPSS) 20.0 (Chicago, IL, USA) software was used to assess statistical significance by the independent samples *t*-test. Differences were considered significant when *P* < 0.05. The number of replicates is indicated in each figure.

## 3. Results

### 3.1. Experiment 1

#### 3.1.1. BD Ameliorates Intestinal Mucosal Injury in OJ Rats

ELISA was performed to measure the serum levels of DAO, IL-1*β*, IL-6, and TNF-*α* in OJ rats. Compared with those in the sham group, IM injury was more severe in the BDL group, and the serum DAO content, and IL-1*β*, IL-6, and TNF-*α* levels were increased in the BDL group (*P* < 0.05). By contrast, rats in the ID group showed a decreased serum DAO content as well as TNF-*α*, IL-6, and IL-1*β* levels compared with those of the BDL group (*P* < 0.05) (Figure 2(a)–2(d)), suggesting that BD can alleviate OJ.

#### 3.1.2. The Autophagic Response of Intestinal Mucosal Cells in OJ Rats Can Be Activated by BD

We next examined the specific mRNA expression of the autophagy markers Beclin-1 and P62 in the intestinal mucosa following bile duct ligation using RT-PCR. Compared with that in the sham group, the expression of Beclin-1 mRNA was downregulated in the IM of BDL rats (*P* < 0.05), whereas the ID group showed upregulated expression of Beclin-1 mRNA compared with that of the BDL group (*P* < 0.05, Figure 3(a)). The Beclin-1 mRNA expression level was increased in the IM of the BDL group. Compared with that of the sham group, the mRNA expression level of the P62 gene in the IM of the BDL group increased (*P* < 0.05, Figure 3(b)). In contrast to that of the BDL group, the P62 mRNA expression level was significantly reduced in the IM of the ID group (*P* < 0.05). These results indicated that BD activates autophagy in OJ rats.

### 3.2. Experiment 2

#### 3.2.1. Autophagy Agonist Ameliorates Intestinal Mucosal Damage in OJ Rats

Rats in the IDR group showed less severe IM damage and decreased serum levels of DAO, IL-1*β*, IL-6, and TNF-*α* compared with those of rats in the ID group (*P* < 0.05, Figure 4(a)–4(d)). The ID3-MA group exhibited decreased indices compared with the ID group (*P* < 0.05, Figure 4(a)–4(d)), indicating that autophagy inhibitors can reduce intestinal mucosal damage in rats with OJ.

#### 3.2.2. Effects of Autophagy Agonist and Inhibitor on Autophagy of the Intestinal Mucosa in OJ Rats Can Be Improved by BD

To further confirm the effects of BD on autophagy in the intestinal mucosa of OJ rats, the mRNA expression of the autophagy markers Beclin-1, LC3, and P62 was detected in the intestinal mucosa of rats after BDL with the administration of RAPA and 3-MA, respectively, using RT-PCR. Compared with the ID group, the RAPA-treated group showed increased mRNA expression levels of the LC3 and Beclin-1 genes (*P* < 0.05, Figure 5(a) and 5(b)) and decreased expression levels of the P62 gene in the IM (*P* < 0.05, Figure 5(c)). Conversely, the ID3-MA group showed decreased expression levels of Beclin-1 and LC3 (*P* < 0.05, Figure 5(a) and 5(b)) and increased P62 mRNA expression levels (*P* < 0.05, Figure 5(c)) compared with those of the ID group. These results showed that BD alleviates intestinal mucosal injury by activating the autophagy pathway in the intestinal mucosa of OJ rats.

#### 3.2.3. Effects of Autophagy Agonist and Inhibitor on Oxidative Stress

To assess the effect of autophagy on oxidative stress in the IM, the levels of ROS, GSH, MDA, and H_2_O_2_ were measured in the rat IM by ELISA. BD significantly increased ROS, MDA, and H_2_O_2_ levels (*P* < 0.05) and decreased GSH levels (*P* < 0.05) in the IM (Figure 6(a)–6(d)). Additionally, compared with those of the ID group, RAPA treatment decreased ROS, MDA, and H_2_O_2_ levels in the rat serum and IM (*P* < 0.05) and increased the GSH level (*P* < 0.05) (Figure 6(a)–6(d)). In addition, the ID3-MA group had increased levels of ROS, MDA, and H_2_O_2_ in both the serum and IM (*P* < 0.05) and decreased levels of GSH (*P* < 0.05) (Figure 6(a)–6(d)) compared with those in the ID group. These results suggested that oxidative stress can be inhibited by the induction of autophagy with BD.

#### 3.2.4. Effect of Autophagy Agonists and Inhibitors on the Activity of Respiratory Chain Complexes

The activity of respiratory chain complex IV significantly increased in the ID group compared with that in the BDL group (*P* < 0.05, Figure 7(a)–7)(e). The RAPA-treated group showed increased activity of respiratory chain complex IV compared with that of the ID group (*P* < 0.05, Figure 7(a)–7)(e). In addition, the ID3-MA group showed decreased respiratory chain complex IV activity compared with that of the ID group (*P* < 0.05, Figure 7(a)–7(e)). These results suggested that mitochondrial damage to the intestinal mucosa can be improved by autophagic responses induced by BD.

## 4. Discussion

The current study revealed that autophagy occurs in OJ and that intraductal BD further induced autophagy and ameliorated intestinal mucosal injury in OJ model rats. After administration of an autophagy agonist, BD increased the occurrence of autophagy in the intestinal mucosa and ameliorated intestinal mucosal injury in OJ rats. When 3-MA was administered, intestinal mucosal injury, oxidative stress, and mitochondrial injury were all aggravated in OJ rats. Therefore, BD can reduce oxidative stress and mitochondrial injury by inducing autophagy in the intestinal mucosa of OJ rats, thereby alleviating intestinal mucosal injury.

The main causes of OJ combined with intestinal mucosal injury are inhibition of Kupffer cells and impaired bacterial clearance induced by hyperbilirubinemia and bile salt deficiency [15]. The degree of damage, as well as the integrity of the intestinal structure, can be reflected by DAO activity, which serves as an ideal indicator of the function of the small intestine. DAO activity is increased upon changes in intestinal permeability and disruption of the intestinal mucosal barrier [16]. Some studies have established an OJ model by ligating the common bile duct, and blood samples were collected to detect DAO activity at 3, 7, and 14 days after surgery; the plasma DAO level was found to increase with prolonged infarct time [17]. Another study showed that plasma DAO levels decreased in OJ rats after they underwent BD [2]. The results of the present study showed that plasma DAO levels decreased following BD, which was consistent with the above findings, indicating that intestinal mucosal injury occurred in OJ rats, which was reduced upon BD. TNF-*α* has a marked effect on the expression of tight junction proteins [2]. IL-1*β* and IL-6 not only regulate the reorganization of cytoskeletal proteins but also directly rearrange tight junction proteins, thus reducing the integrity of the barrier [18]. Proinflammatory cytokines such as TNF-*α*, IL-1*β*, and IL-6 are highly expressed in response to OJ [19, 20]. However, this inflammation could be attenuated by BD. In particular, BD decreases bile accumulation and reduces the inflammatory response, which in turn decreases the levels of IL-1*β*, IL-6, and TNF-*α*.

Autophagy helps to increase the adaptive capacity of cells in response to a variety of adverse stimuli and plays an important role in the renewal of the intracellular environment and maintenance of homeostasis in vivo [21]. Autophagy is closely related to inflammation. Inflammatory responses can be modulated by multiple signaling pathways of autophagy, and cytokines can regulate autophagic responses [22, 23]. The present data showed that an autophagy activator (RAPA) attenuated inflammation in the intestinal mucosal tissues; however, inflammation was further exacerbated by treatment with an autophagy inhibitor (3-MA).

ROS are produced under physiological conditions and are critical for the maintenance of cellular activities. However, excessive ROS production or aggregation can cause serious damage [24]. ROS-induced MDA and H_2_O_2_ are considered to be indicators of cytotoxicity [25]. The main antioxidant of the cellular defense system is GSH, which acts during oxidative stress by being converted into oxidized glutathione (GSSG) [26]. Previous studies have shown that oxidative damage occurring in intestinal mucosal cells is mainly caused by OJ [27]. The present data showed that OJ can lead to increased levels of oxidative stress, including ROS, MDA, and H_2_O_2_ and decreased levels of GSH. RAPA attenuated oxidative damage in the intestinal mucosal tissues of OJ rats, and the degree of oxidative damage was further exacerbated by 3-MA. These results showed that autophagy is an important factor in attenuating oxidative damage in intestinal injury induced by OJ.

ROS are byproducts of the energy-producing processes of the mitochondrial respiratory chain [28]. Deficient or impaired antioxidant activity in the cell will cause the excessive accumulation of ROS in the mitochondria because they cannot be eliminated, which eventually leads to the development of mitochondrial dysfunction and even oxidative stress-related injury [29]. The mitochondrial respiratory chain consists of primary and secondary respiratory chains, with the primary respiratory chain consisting of complexes I, III, and IV, and the secondary respiratory chain consisting of complexes II, III, and IV, with complex V being an ATP synthase [30]. A previous study showed that the intestinal mucosal damage that occurs in OJ is primarily due to mitochondrial damage, and the induction of cellular autophagy promotes the recovery of mitochondrial function [31]. In the present study, the activity of active complex IV of the mitochondrial respiratory chain was decreased in OJ model rats, and the assay results suggested that mitochondrial function was impaired. The activity level of complex IV of the mitochondrial respiratory chain was increased following BD, and mitochondrial function in the intestinal mucosa was strengthened when autophagy agonists were administered to the ID group, whereas the degree of mitochondrial damage was more severe in the presence of 3-MA. These findings suggest that autophagy plays a key role in the alleviation of mitochondrial damage induced by OJ following BD.

The main limitations of this study are that the pathways regulating autophagy were not investigated further, and a control group for external BD was not established owing to the limited number of animals used.

In conclusion, this study revealed that autophagy occurs in the intestinal mucosa of OJ rats and that BD enhances the level of autophagy. These results suggest that intra-BD may reduce the inflammatory response, oxidative damage, and mitochondrial injury by modulating intestinal mucosal autophagy.

## Figures and Tables

**Figure 1:** Experimental flowchart. Sham: no bile duct ligation; BDL: bile duct ligation; ID: internal drainage; IDR: internal drainage + rapamycin; ID3-MA: internal drainage  +  3-methyladenine.

**Figure 2:** Intrabiliary drainage attenuates the inflammatory response and ameliorates intestinal mucosal injury in rats with obstructive jaundice. (a) Serum TNF-*α*, (b) IL-6, (c) IL-1*β*, and (d) DAO levels. Data are expressed as means ± SEM (*n* = 10). Sham: no bile duct ligation; BDL: bile duct ligation; ID: internal drainage; TNF-*α*: tumor necrosis factor-*α*; IL-6: interleukin-6; IL-1*β*: interleukin-1*β*; DAO: diamine oxidase. a: P < 0.05 vs. sham group. b: P < 0.05 vs. BDL group.

**Figure 3:** Autophagy response of intestinal mucosal cells in rats with obstructive jaundice can be activated by intrabiliary drainage. The expression levels of autophagy-related genes were detected by RT-PCR. (a) Beclin-1 mRNA expression levels. (b) P62 mRNA expression levels. Data are expressed as means ± SEM (*n* = 10). Sham: no common bile duct ligation; BDL: bile duct ligation; ID: internal drainage; a: *P* < 0.05 vs. sham group. b: *P* < 0.05 vs. BDL group.

**Figure 4:** Effects of autophagy agonist and inhibitor on intestinal mucosal injury in obstructive jaundice model rats with biliary drainage. (a) Serum TNF-*α*, (b) IL-6, (c) IL-1*β*, and (d) DAO levels. Data are expressed as means ± SEM (*n* = 10). BDL: bile duct ligation; ID: internal drainage; IDR: internal drainage + rapamycin; ID3-MA: internal drainage  +  3-methyladenine. TNF-*α*: tumor necrosis factor-*α*; IL-6: interleukin-6; IL-1*β*: interleukin-1*β*; DAO: diamine oxidase. a: *P* < 0.05 vs. BDL group. b: *P* < 0.05 vs. ID group. c: *P* < 0.05 vs. IDR group.

**Figure 5:** Effects of autophagy agonist and inhibitor on autophagy in obstructive jaundice model rats with biliary drainage. RT-PCR was used to detect the expression levels of autophagy-related genes. (a) Beclin-1 mRNA expression levels. (b) LC3I mRNA expression levels. (c) P62 mRNA expression levels. BDL: bile duct ligation; ID: internal drainage; IDR: internal drainage + rapamycin; ID3-MA: internal drainage  +  3-methyladenine. a: *P* < 0.05 vs. BDL group. b: *P* < 0.05 vs. ID group. c: *P* < 0.05 vs. IDR group.

**Figure 6:** Effects of autophagy agonist and inhibitor on intrabiliary drainage on oxidative stress in the intestinal mucosal cells of obstructive jaundice model rats. (a) Serum ROS, (b) MDA, (c) H_2_O_2_, and (d) GSH levels, (e) tissue ROS, (f) tissue MDA, (g) tissue H_2_O_2_, and (h) tissue GSH levels. Data are expressed as means ± SEM (*n* = 10). BDL: bile duct ligation; ID: internal drainage; IDR: internal drainage + rapamycin; ID3-MA: internal drainage  +  3-methyladenine; ROS: reactive oxygen species; MDA: malondialdehyde; H_2_O_2_: hydrogen peroxide; GSH: glutathione. a: *P* < 0.05 vs. BDL. b: *P* < 0.05 vs. ID. c: *P* < 0.05 vs. IDR.

**Figure 7:** Effects of autophagy agonist and inhibitor on the activity of respiratory chain complexes I–Vin the mitochondria of intestinal mucosal cells of rats with obstructive jaundice. Data are expressed as means ± SEM (*n* = 10). BDL: bile duct ligation; ID: internal drainage; IDR: internal drainage + rapamycin; ID3-MA: internal drainage  +  3-methyladenine. a: *P* < 0.05 vs. BDL. b: *P* < 0.05 vs. ID. c: *P* < 0.05 vs. IDR.

**Table 1:** Primer sequence.

Gene		Primer sequence
Beclin-1	Forward primer	5′-CGTGGAGAAAGGCAAGATT-3′
	Reverse primer	5′-AGAACTGTGAGGACACCCAAG-3′

LC3	Forward primer	5′-GACCCTCTACGATGCTGGTG-3′
	Reverse primer	5′-TGCTGTCCTCAATGTCCTTCT-3′

P62	Forward primer	5′-CTGCTGCCTCCCTCTAATCC-3′
	Reverse primer	5′-TATTCTCCGGCTCCATCTTG-3′

*β*-Actin	Forward primer	5′-CATTGCTGACAGGATGCAGAAG-3′
	Reverse primer	5′-GAGCCACCAATCCACACAGAGT-3′

## Data Availability

The datasets used and analyzed during the current study are available from the corresponding author upon reasonable request.
